# Investigating the Role of Image Fusion in Brain Tumor Classification Models Based on Machine Learning Algorithm for Personalized Medicine

**DOI:** 10.1155/2022/7137524

**Published:** 2022-02-07

**Authors:** R. Nanmaran, S. Srimathi, G. Yamuna, S. Thanigaivel, A. S. Vickram, A. K. Priya, Alagar Karthick, J. Karpagam, V. Mohanavel, M. Muhibbullah

**Affiliations:** ^1^Department of Biomedical Engineering, Saveetha School of Engineering, Saveetha Institute of Medical and Technical Sciences, Saveetha University, Chennai, 602105 Tamil Nadu, India; ^2^Department of Electronics and Communication Engineering, Faculty of Engineering and Technology, Annamalai University, Annamalainagar, 608002 Tamil Nadu, India; ^3^Department of Biotechnology, Saveetha School of Engineering, Saveetha Institute of Medical and Technical Sciences, Saveetha University, Chennai, 602105 Tamil Nadu, India; ^4^Department of Civil Engineering, KPR Institute of Engineering and Technology, Coimbatore, 641407 Tamil Nadu, India; ^5^Department of Electrical and Electronics Engineering, KPR Institute of Engineering and Technology, Coimbatore, 641407 Tamil Nadu, India; ^6^Centre for Materials Engineering and Regenerative Medicine, Bharath Institute of Higher Education and Research, Chennai, 600073 Tamil Nadu, India; ^7^Department of Electrical and Electronic Engineering, Bangladesh University, Dhaka 1207, Bangladesh

## Abstract

Image fusion can be performed on images either in spatial domain or frequency domain methods. Frequency domain methods will be most preferred because these methods can improve the quality of edges in an image. In image fusion, the resultant fused images will be more informative than individual input images, thus more suitable for classification problems. Artificial intelligence (AI) algorithms play a significant role in improving patient's treatment in the health care industry and thus improving personalized medicine. This research work analyses the role of image fusion in an improved brain tumour classification model, and this novel fusion-based cancer classification model can be used for personalized medicine more effectively. Image fusion can improve the quality of resultant images and thus improve the result of classifiers. Instead of using individual input images, the high-quality fused images will provide better classification results. Initially, the contrast limited adaptive histogram equalization technique preprocess input images such as MRI and SPECT images. Benign and malignant class brain tumor images are applied with discrete cosine transform-based fusion method to obtain fused images. AI algorithms such as support vector machine classifier, KNN classifier, and decision tree classifiers are tested with features obtained from fused images and compared with the result obtained from individual input images. Performances of classifiers are measured using the parameters accuracy, precision, recall, specificity, and *F*1 score. SVM classifier provided the maximum accuracy of 96.8%, precision of 95%, recall of 94%, specificity of 93%, *F*1 score of 91%, and performed better than KNN and decision tree classifiers when extracted features from fused images are used. The proposed method results are compared with existing methods and provide satisfactory results.

## 1. Introduction

Early detection of cancer plays a vital role in the healthcare industry because when abnormal tissue or cancer is found early, it is easy to plan successful treatment [1, 2]. If cancer spreads to neighbor cells, it is challenging to treat, and survival chances are much lower. Many machine learning techniques were developed to detect cancer at early stages [3, 4]. Still, a tool with more accuracy and less processing time is needed. This research is aimed at detecting cancer irrespective of its types by combining two imaging modalities, such as CT/PET or MRI/SPECT, which provides better accuracy than existing methods. Finally, the concept is extended to cancer classification to predict the tumor type, whether it belongs to benign or malignant tumors [5, 6]. While there are many studies in image fusion for the visual enhancement of images, very few types of research focus on the influence of image fusion in other applications such as image classification. The role of image fusion in remote sensing is significant, and almost every recent sensor development for earth applications considers channels with different spatial resolutions [7, 8]. Image fusion improves the information content by combining two or more images using a specific algorithm [3]. A case study on the influence of image fusion approaches on classification accuracy for remote sensing applications is more relevant to this research work. They took Landsat 7 ETM+ image for the analysis. They analyzed various image fusion approaches such as adaptive image fusion (AIF), wavelet-based fusion, multisensor multiresolution fusion technique (MMT), principal component analysis (PCA), hue saturation-value transform (HSV), and Brovey method of fusion. The fusion results were employed for maximum likelihood classifier, object-based classification, and support vector machine classifier [9]. The Brovey Transform (BT) was created to visually boost contrast between the image histogram's low and high ends. BT produce the spectral degradation, which should not be employed if the original scene radiometry must be preserved. Brovey Transform resulted in low dynamic range resultant image and significant misclassification detected when using pixel-based classifiers. HSV fusion was not assigning the discrete classes from the training dataset. Another method called principal component analysis performed better because of its capability of separately high- and low-frequency parts of an image. MMT fusion technique produced “Speckle” noise in the classification, which results in poor edge detection. They concluded in the case study that wavelet transform-based fusion improves the classification accuracy, and they recommended the classification application. Wavelet transforms are used to portray abrupt peaks and discontinuities. Wavelet transform has a number of drawbacks, including shift sensitivity and directional selectivity [10, 11].

The research on the effects of image fusion algorithms on classification accuracy in remote sensing applications was conducted. They took Quickbird-02 panchromatic and multispectral images over the city of Wuhan (China) and analyzed the effects of fusion on unsupervised ISODATA (iterative self-organizing data analysis) classifier accuracy. They considered eight image fusion techniques and analyzed the effects of fusion on improving classification accuracy. They found that the high pass filter-based fusion method performs worst because of its injection of high-frequency information [12]. They concluded that the region-based image fusion method improves the accuracy of the classifier. Even though colour distortion occurs, the contrast of the fused image is higher, which is very helpful in interpretation and classification, and they recommended a region-based fusion technique for classification application. Region-based image fusion has several advantages over pixel-based image fusion methods, such as being less susceptible to noise, more resilient, and avoiding misregistration, but it is also more difficult.

Kumar et al. have proposed a novel MSLN-CNN method to solve the HSI classification problems, multilayer spatial-spectral feature fusion and sample augmentation with local and nonlocal constraints (MSLN-CNN). The authors make full use of complementary spatial-spectral information among different layers, and compared with other deep learning models, CNN has two unique structures: local connection and weight sharing. The representative classifiers include *k*-nearest neighbors, logistic regression, support vector machine (SVM), sparse representation-based classification, and extreme learning machine [13, 14]. Among these classifiers, SVM seeks to separate the samples with different classes. Finally, the authors concluded that MSLN-CNN could achieve end-to-end classification by optimizing multilayer spatial-spectral feature fusion jointly. It is a promising method to deal with the overfitting problem by considering local spatial and nonlocal spectral constraints.

Chandran et al. have developed an approach for fusing features obtained from multisensor compressive measurements for spectral image classification. This fusion method merged the components extracted from data captured by sensors that satisfy the Nyquist–Shannon sampling theorem. They developed a low-resolution feature as degraded versions of the high-resolution features [15]. Also, they formulated an inverse problem that aims at estimating high-resolution characteristics, including both a sparsity-inducing term and a total variation (TV) regularization term to exploit the correlation between neighboring pixels of the spectral image. Therefore, they improved the performance of pixel-based classifiers. Besides, they introduce the mathematical model of the high-resolution features. This model describes the relationship between the high-resolution elements and the spectral image under test. The authors described an algorithm based on the alternating direction method of multipliers (ADMM) for solving the fusion problem. The proposed feature fusion approach is tested for two CSI architectures: three-dimensional coded aperture snapshot spectral imaging (3D-CASSI) and colored CASSI (C-CASSI). Finally, they compared the proposed feature fusion method concerning state-of-the-art feature extraction and fusion techniques which improves the accuracy and robustness to noise [16, 17]. They concluded that the ADMM algorithm performs better when compared to existing methods. Because of its fast convergence speed in many applications, the ADMM technique has sparked a lot of academic attention in recent years.

Most of the related research was attempted only in remote sensing, focusing on medical imaging applications. Based on the above literature, many researchers reported that image fusion could improve image quality, and no research analyzes with experiment results. This research work shows how image fusion improves the visual quality of medical images and how these images further improve classification accuracy with experiment results. This research work combines brain tumor images from MRI and SPECT modalities using the discrete cosine transform (DCT) method. The magnetic resonance interference (MRI) imaging technique can produce incredibly detailed diagnostic images of most of body's major organs and tissues that other imaging techniques cannot. Because MRIs do not involve radiation, they are safe for children and pregnant people to undergo. The SPECT (single-photon emission computed tomography) imaging technology can be used to determine whether or not there is enough blood flow to various parts of the brain. SPECT scans can be used to acquire data on changes in brain function as a result of disease. Benefits of two imaging modalities can be attained in a single image when these two modalities are merged. The fused image provides more information to the doctors than the individual input images. Apart from that, when compared to individual input images, the number of features or attributes recovered from fused images is higher. As a result, cancer classification will be more precise, allowing doctors and other health care providers to better plan therapy for their patients. In order to combine MRI and SPECT images, discrete cosine transform-based image fusion technique has developed with improved fusion parameters such as peak signal to noise ratio (PSNR), structural similarity index measure (SSIM), and normalized correlation (NC). High values of PSNR in dB, SSIM in %, and NC in % indicates improved fusion between two images. This proposed DCT-based fusion technique provides high PSNR, SSIM, and NC which is used for fusing MRI and SPECT images in this research work.

Three classifiers, namely, support vector machine, *K*-nearest neighbour classifier, and decision tree classifiers, are used in this research work to classify the brain tumour images into benign or malignant classes. The performance of these classifiers is measured and compared based on accuracy, precision, recall, specificity, and *F*1 score. In order to analyze the effect of image fusion, the experiment results are compared with the result obtained when MRI input image alone was used, SPECT input image alone was used for classification. Algorithms of all these three classifiers are explained in the “Research Methods” section, and the performance metrics are explained in the next section.

## 2. Research Methods

The proposed brain tumour classification model is shown in Figure 1.The input images such as MRI and SPECT images are collected from http://kaggle.com for analysis. Image registration was applied to input images before applying the image fusion method. Image fusion using discrete cosine transform was developed, and fused images were obtained. Thirty features were extracted from fused images, and they were given as input to three classifiers. Classifier's performance is measured using accuracy, precision, recall, specificity, and *F*1 score. These results were compared with the classifier results when features extracted from individual input images were given to the classifiers. High values of performance metrics indicate the better performance of classifiers.

### 2.1. Preprocessing of Brain Tumour Images

The visual quality of input medical images such as MRI and SPECT images are improved by applying contrast limited adaptive histogram equalization (CLAHE) technique [18, 19]. Instead of operating on entire image pixels, CLAHE operates only on a small region of the image called tiles [20, 21]. Image registration needs to be applied before applying the image fusion technique. A parametric transformation Ta(.) is applied to the target image to maximize the similarity between the target image and the reference image to make it similar to *I*_*r*_ [22]. The optimization target can be represented as in Equation (1).

(1) $$\begin{array}{c} \text{Ta}\left(.\right)=\arg\max\rho \left({\text{I}}_{\text{r},}\right.{\text{T}}_{\text{a}}\left({\text{I}}_{\text{t}}\right). \end{array}$$

Various steps involved in image registration include similarity measure, point detection and extraction, applying image descriptors, point selection, pattern matching, image resampling, and compositing [23].

### 2.2. Image Fusion Using Discrete Cosine Transform

Fusion can be performed in spatial or frequency-domain methods, and DCT belongs to the frequency domain category. When DCT is applied to input images, it decomposes the images into DCT coefficients, and in the transform domain, the fusion rules are applied [24–26]. After applying inverse DCT, a fused image is obtained in the spatial domain [27, 28]. Input images such as MRI and SPECT images are applied with discrete cosine transform, which provides DCT coefficients, and averaging fusion rule is applied in the frequency domain, which provides fused DCT coefficients. Inverse discrete cosine transform is applied on fused DCT coefficients to obtain fused images at spatial domain [25, 29–32]. Image fusion using discrete cosine transform is shown in Figure 2.

Discrete cosine transform of two-dimensional image *X*(*n*_1_, *n*_2_) of size *M* × *N* is represented by Equation (2). Here, *M* represents number of rows in an image, and *N* represents number of columns in an image.

(2) $$\begin{array}{c} X\left(k_{1},k_{2}\right)=\overset{M-1}{\underset{n_{1}=0}{\sum }}\overset{N-1}{\underset{n_{2}=0}{\sum }}x\left(n_{1},n_{2}\right)\cos\left(\frac{\pi \left(2n_{1}+1\right)k_{1}}{2M}\right)\cos\left(\frac{\pi \left(2n_{2}+1\right)k_{2}}{2N}\right), \end{array}$$

where *n*_1_, *n*_2_ are the spatial domain coordinates and *k*_1_, *k*_2_ are the frequency domain coordinates.

Similarly, inverse discrete cosine transform of two-dimensional image *X* (*k*_1_, *k*_2_) of size *M* × *N* is represented by

(3) $$\begin{array}{c} X\left(k_{1},k_{2}\right)=\overset{M-1}{\underset{k_{1}=0}{\sum }}\overset{N-1}{\underset{k_{2}=0}{\sum }}x\left(k_{1},k_{2}\right)\cos\left(\frac{\pi \left(2n_{1}+1\right)k_{1}}{2M}\right)\cos\left(\frac{\pi \left(2n_{2}+1\right)k_{2}}{2N}\right), \end{array}$$

where *k*_1_ ranges from 0 to *M* − 1 and *k*_2_ ranges from *N* − 1.

### 2.3. Support Vector Machine Classifier

SVM classifiers are supervised learning methods that are used for regression and classification.

The SVM classifier can maximize the geometric margin and minimize the classification error, and hence, the SVM classifier can also be called maximum margin classifiers [33–40]. SVM classifiers are not biased by outliers and not sensitive to overfitting but they are not suitable when huge number of features used and for nonlinear problems.

Let us consider a dataset (*A*_1_, *B*_1_, ..*A*_*n*_, *B*_*n*_), where (*A*_1_, *A*_2_..*A*_*n*_) is the set of the input variable, (*B*_1_, *B*_2_.., *B*_*n*_) is the output variable, and ‘*C*' is the intercept, then the SVM classifier is given as in

(4) $$\begin{array}{c} \text{SVM}=\overset{i}{\underset{m=1}{\sum }}\beta_{m}-\frac{1}{2}\overset{i}{\underset{m,n=1}{\sum }}b_{m}b_{n}C\left(a_{m},a_{n}\right)\beta_{m}\beta_{n}, \end{array}$$

where *m* = 1, 2, 3 ⋯ .*i* and *C* = *b*_*m*_*β*_*m*_ + *b*_*n*_*β*_*n*_.

### 2.4. *K*-Nearest Neighbour Classifier

*K*-nearest neighbor classification is more suitable for large datasets, and it takes more computation time for testing than training the dataset. The *K*-nearest neighbor classification technique is the most straightforward technique that provides good classification accuracy and stability [41, 42]. The *K*-NN algorithm is based on distance functions such as Manhattan, Minkowski, Tanimoto, Jaccard, Mahalanobis, and Euclidean distance in which Euclidean distance is more common [43, 44]. It is mathematically given in

(5) $$\begin{array}{c} d\left(a,b\right)=\sqrt{\overset{m}{\underset{i=1}{\sum }}{\left(b_{i-}\;a_{i}\right)}^{2}}, \end{array}$$

where

*a*, *b* = Two points in Euclidean distance

*a*_*i*_, *b*_*i*_ = Euclidean Vectors

*m* = *m*-space.

Even though the KNN classifier runs slowly, its computational power is more. KNN algorithm consists of the training phase and testing phase. Features or attributes are stored during the training phase, and while in the testing phase, the features from testing images are compared with stored features, and the class will be determined [45].

*K*-NN algorithm consists of the following steps:

1. Determine suitable distance metrics like Euclidean distance
2. Store all the training datasets in the training phase
3. During the testing phase, compute the distances between the new feature and stored features
4. The correct classification access given in the test phase is used to assess the correctness of the algorithm

### 2.5. Decision Tree Classifier

A decision tree is a supervised learning technique that can be used for both regression and classification problems, but it is mainly used for classification problems. Decision tree classifiers are appropriate for both linear and nonlinear systems; however, they are ineffective when dealing with limited datasets. In a decision tree classifier, overfitting is a common occurrence. Nodes in the tree-like structure represent the features of a dataset, branches represent the decision rules, and leaf node represents the output [46, 47]. The decision trees usually resemble human thinking ability; hence, it is easy to understand. The algorithm starts at the root node and compares the attributes of root nodes with attributes of record nodes. Based on the comparison, it jumps to the next node. Many algorithms are proposed for learning decision tree from a given dataset, but commonly, ID3 algorithm is preferred due to its simplicity for implementation [48–51]. ID3 algorithm is a top-down greedy search of possible branches, and it uses information gain and entropy to build the tree.

The *H*(*Y*) Shannon entropy of a random discrete variable *Y* with possible *Y*_1_, *Y*_2_ ⋯ .*Y*_*n*_ and probability mass function *P*(*Y*) is defined as in

(6) $$\begin{array}{c} H\left(Y\right)=-\overset{n}{\underset{i=1}{\sum }}P\left(y_{i}\right)\log_{2}P\left(y_{i}\right). \end{array}$$

Entropy is equal to zero for a completely homogeneous dataset, and entropy is equal to one of the datasets equally divided. A branch with entropy more than one needs splitting.

### 2.6. Experimental Setup

MATLAB version 2021 software is used for this research work. Proposed work consists of steps such as preprocessing, image fusion, feature extraction, and image classification. For preprocessing using CLAHE, DCT-based image fusion technique and feature extraction MATLAB script have developed, and result is obtained. For testing with different classifiers and analysis, MATLAB inbuilt classification learner application is used. The result which obtained feature extraction is stored in excel file, and this file is directly given as input to classification learner application in order to analyze the effect of image fusion on SVM, *K*-NN, and decision tree classifiers.

## 3. Results and Discussion

### 3.1. Comparison of Our Method with KNN Classifier and Decision Tree Classifier

Input images such as brain tumors from CT modality and SPECT modality are shown in Figures 3(a) and 3(b), respectively. A converted grayscale image of SPECT image is shown in Figure 3(c). After applying with CLAHE for image enhancement and registration, the two input images are applied with DCT-based image fusion technique and the resultant fused image Figure 3(d).

Two hundred MRI images and 200 SPECT images are fused, providing 200 fused images. Features such as radius, area, perimeter, texture, smoothness, compactness, concave points, and concavity are considered, and thus, six features in total are extracted from fused images and individual input images such as MRI and SPECT images. A scatter plot representing some of the features is shown in Figure 4. These features are given as input to SVM, KNN, and decision tree classifiers, and the results are compared to identify the best classifier for brain tumor detection.

The performances of classifiers are measured using accuracy, precision, recall, specificity, *F*1 score, confusion matrix, and ROC curve. The confusion matrix typically consists of four different results, namely, true positive (TP), false positive (FP), true negative (TN), and false negative (FN). Performance measures of classifiers are described in this section.

### 3.2. Accuracy

The accuracy of the classifier is defined as the ratio of total number of correct predictions to the total number of predictions. Accuracy is defined in Equation (7), as shown below.

(7) $$\begin{array}{c} \text{Accuracy}=\frac{\text{TP}+\text{TN}}{\text{TP}+\text{TN}+\text{FN}+\text{FP}}. \end{array}$$

### 3.3. Precision

The precision of the classifier is defined as the correct prediction ratio to the actual prediction of brain tumor cases represented

(8) $$\begin{array}{c} \text{Precision}=\frac{\text{TP}}{\text{TP}+\text{FP}}. \end{array}$$

### 3.4. Recall

Recall of the classifier is defined as the ratio of correctly predicted brain tumor cases to overall brain tumor cases, including nonbrain tumor cases. The recall is defined in

(9) $$\begin{array}{c} \text{Recall}=\frac{\text{TP}}{\text{TP}+\text{FN}}. \end{array}$$

### 3.5. Specificity

The specificity of the classifier is defined as the ratio of correctly identified nonbrain tumor cases to negative brain tumor cases, which is represented as in

(10) $$\begin{array}{c} \text{Specificity}=\frac{\text{TN}}{\text{TN}+\text{FP}}. \end{array}$$

### 3.6. *F*1 Score

It is the measure of average between precision and recall of classifiers defined in

(11) $$\begin{array}{c} F1\text{ Score}=\frac{\text{Precision}\times \text{Recall}}{\text{Precision}+\text{Recall}}. \end{array}$$

### 3.7. Confusion Matrix

The performance of the classifier in matrix form is given by the confusion matrix of the prediction model. It consists of correctly identified brain tumor cases, missclassified brain tumor results, correctly identified nontumor cases, and missclassified nonbrain tumor cases.

### 3.8. Receiver-Operating Characteristic (ROC)

The ROC curve graph graphically illustrates the performance of the classifier. This graph shows the relationship between the actual positive rate and the false-positive rate.

Extracted features from fused images are tabulated and plotted using parallel coordinates plot as shown in Figure 5.

The confusion matrix of the SVM classifier, *K*-NN classifier, and decision tree classifier is shown in Figures 6(a)–6(c), respectively. Performance measures such as accuracy, precision, recall, specificity, and *F*1 score for SVM, KNN, and decision tree classifiers are tabulated in Table 1.

The classifiers are stored with extracted feature values during training phase. During testing phase, classifiers are tested with different input images. Initially, the classifiers are tested with cancerous input images. If the classifier predicts the cancerous image output correctly, this condition can be taken as true positive (TP) but if it is wrongly predict as noncancerous image, then the condition is known as false positive (FP). When the classifiers are tested with noncancerous input images, if the classifier predicts the noncancerous image output correctly, this condition can be taken as true negative (TN) but if it is wrongly predict as cancerous image, then the condition is known as false negative (FN). Based on this TP, FP, TN, and FN values obtained from confusion matrix as shown in Figures 6(a)–6(c), the performance measures of classifiers are calculated using Equations (7) to (11) and tabulated as shown in Table 1.

From tabulated results, it is inferred that the SVM classifier provides high accuracy, precision, recall, specificity, and *F*1 score parameters and thus performs better than *K*-NN and decision tree classifier.

The performance of classifiers can also be predicted using the response of the ROC curve based on the value of the area under the curve. The area under curve values of the SVM, KNN, and decision tree classifier is 0.994, 0.932, and 0.921, as shown in Figures 7(a)–7(c). From observation, it is noted that the SVM classifier gives the maximum area under the curve value of 0.994, which indicates the better performance of the classifier over the other two classifiers.

### 3.9. Comparison of Our Method with Features Extracted From MRI Image Alone Given as Input to Classifiers

Features are extracted from 200 samples of MRI images collected from the medical database, and these features are given as input to SVM, KNN, and decision tree classifiers. The results of classifiers are tabulated in Table 2.

From tabulated results, it is inferred that SVM classifier when fused images are considered for feature extractions provides an accuracy of 96.3%, the precision of 97.5%, recall of 95.12%, specificity of 97.13%, and F1 score of 96.29%. These five parameters are high values and thus perform better than SVM, *K*-NN, and decision tree classifiers when MRI image alone is considered for feature extraction.

### 3.10. Comparison of Our Method with Features Extracted From SPECT Image Alone Given as Input to Classifiers

Features are extracted from 200 SPECT images collected from a medical database, and these features are given as input to SVM, KNN, and decision tree classifiers. The results of classifiers are tabulated in Table 3.

From tabulated results, it is inferred that SVM classifier when fused images are considered for feature extractions provides an accuracy of 96.8%, the precision of 97.5%, recall of 95.12%, specificity of 97.13%, and *F*1 score of 96.29%. These five parameters are high values and thus perform better than SVM, *K*-NN, and decision tree classifiers when SPECT image alone is considered for feature extraction.

### 3.11. Comparison of Our Method with SVM, KNN Classifier, and Decision Tree Classifier In Terms of Consumed Time

In this test, we compare the implementation time of our proposed method and SVM, KNN, and decision tree classifiers when features from SPECT image alone are given as input to classifiers, and the obtained result is shown in Table 4.

Ten independent experiments are taken on PC with Intel Core 3 processor and PC with Celeron 3.06G/1G processor, and the average time is calculated. From the tabulated results, it is observed that the proposed SVM classifier when features from fused images are given as input to classifier consumes longer time, almost 420 seconds, to execute the results, whereas SVM, KNN, and decision tree classifiers when features from SPECT image alone given as input to classifier consume 128, 160, and 180 seconds, respectively. The existing methods involve steps like preprocessing, feature extraction, segmentation, and classification, whereas the proposed method involves steps like preprocessing, image fusion, feature extraction, segmentation, and classification. Because of the additional step involved, the proposed method consumes more time to execute the results when compared to existing research methods. The experiment results of the proposed method are compared with relevant literature and presented in Table 5.

## 4. Conclusion

Brain tumor images from MRI and SPECT modalities are considered and applied with CLAHE method to preprocess the images, and then, DCT-based fusion technique was applied to obtain fused images. Features from fused images are extracted and inputted to SVM, KNN, and the decision tree classifier. SVM classifier provides the maximum accuracy of 96.8%, precision of 97.5%, recall of 95.12%, sensitivity of 97.43%, and *F*1 score of 96.29%, which is higher when compared to SVM, KNN, and decision tree classifier when features from either MRI or SPECT image is alone given as input to classifiers. As this research involved image fusion and preprocessing feature extraction and image classification, it took a long time to execute the results compared to conventional cancer classification models. These novel fusion-based AI algorithms can be more suitable for personalized medicine. In the future, transform-based image fusion approaches such as Curvelet transform and Shearlet transform can be applied to input images, and the classification performance can be measured.

## Figures and Tables

**Figure 1:** Proposed fusion-based brain tumor classification model.

**Figure 2:** Discrete cosine transform-based image fusion methodology.

**Figure 3:** (a) Input image-1 (MRI-brain tumor. (b) Input image-2 (SPECT-brain tumor. (c) Converted grey scale image of input image-2. (d) Fused image (MRI-SPECT).

**Figure 4:** (a) Scatter plot representation of mean perimeter and mean area. (b) Scatter plot representation of mean smoothness and mean compactness. (c) Scatter plot representation of standard error mean concavity and standard error mean concave points. (d) Scatter plot representation of worst symmetry and worst fractal dimension.

**Figure 5:** Parallel coordinates plot of features extracted from malignant type tumor.

**Figure 6:** (a) Confusion matrix of the SVM classifier. (b) Confusion matrix of the *K*-NN classifier. (c) Confusion matrix of the decision tree classifier.

**Figure 7:** (a) ROC curve of the SVM classifier. (b) ROC curve of the KNN classifier. (c) ROC curve of the SVM classifier.

**Table 1:** Performance measures of SVM, KNN, and decision tree classifiers when features extracted from fused images are given as input.

S. no.	Classifier name	TP	FP	TN	FN	Accuracy	Precision	Recall	Specificity	*F*1 score
1	SVM	195	5	190	10	96.8	97.5	95.12	97.43	96.29
2	*K*-NN	186	14	187	13	93.3	93	93.46	93.03	93.23
3	Decision tree	181	19	182	18	90.8	90.5	90.95	90.54	90.72

**Table 2:** Performance comparison of proposed method and SVM, KNN, and decision tree classifiers when MRI image alone given as input.

S. no.	Classifier name	TP	FP	TN	FN	Accuracy	Precision	Recall	Specificity	*F*1 score
1	SVM (proposed)	195	5	190	10	96.8	97.5	95.12	97.43	96.29
2	SVM	190	10	186	14	94	95	93.21	94.89	94.09
3	*K*-NN	180	20	181	19	90.25	90	90.45	90.04	90.20
4	Decision tree	174	26	172	28	86.50	87	86.86	86	87

**Table 3:** Performance comparison of proposed method and SVM, KNN, and decision tree classifiers when SPECT image alone given as input.

S. no.	Classifier name	TP	FP	TN	FN	Accuracy	Precision	Recall	Specificity	*F*1 score
1	SVM (proposed)	195	5	190	10	96.8	97.5	95.12	97.43	96.29
2	SVM	192	8	188	12	95	96	94.11	95.91	95.04
3	*K*-NN	182	18	185	15	91.75	91	92.38	91.13	91.68
4	Decision tree	178	22	179	21	89.25	89	89.44	89.05	89.21

**Table 4:** Performance comparison of proposed method and SVM, KNN, and decision tree classifier based on consumed time.

Parameter	Classifiers			
	SVM (proposed)	SVM	*K*-NN	Decision tree
Time consumed (seconds)	420	128	160	180

**Table 5:** Comparison of our method with existing methods from literature.

Reference	Classifiers name	Accuracy (%)	Sensitivity (%)	Precision (%)
Present study	SVM, KNN, decision tree	96.80	97.43	97.5
Masoudi S et al. 2021 [52]	Resnet-101C	86.3	NA	NA
Welikala RA et al. 2020 [53]	R-CNN	NA	89.51	84.77
Anupama et al. 2019 [54]	CNN-capsule network	92.5	93	96
T Nguyen et al. 2019 [55]	CNN	73.68	NA	NA
Erkal B et al. 2020 [56]	Multilayer perceptron	97	NA	NA

## Data Availability

The data used to support the findings of this study are included in the article.

## References

[1] Pohl C., Van Genderen J. L. (1998). Review article multisensor image fusion in remote sensing: concepts, methods and applications. *International journal of remote sensing*.

[2] Pohl C., van Genderen J. L. (1994). Multisensor fusion: optimization and operationalization for mapping applications. *Signal Processing, Sensor Fusion, and Target Recognition III*.

[3] Colditz R. R., Wehrmann T., Bachmann M. (2006). Influence of image fusion approaches on classification accuracy: a case study. *International Journal of Remote Sensing*.

[4] ME V., DR V., MK M., MP S. (2018). A novel technique for optimizing panchromatic and multispectral image fusion using discrete wavelet transform. *International Journal of Engineering and Technology*.

[5] Sara D., Mandava A. K., Kumar A., Duela S., Jude A. (2021). Hyperspectral and multispectral image fusion techniques for high resolution applications: a review. *Earth Science Informatics*.

[6] Feng X., He L., Cheng Q., Long X., Yuan Y. (2020). Hyperspectral and multispectral remote sensing image fusion based on endmember spatial information. *Remote Sensing*.

[7] Yuhendra A. I., Sri Sumantyo J. T., Kuze H. (2011). Spectral quality evaluation of pixel-fused data for improved classification of remote sensing images. *IEEE International Geoscience and Remote Sensing Symposium*.

[8] Singh R., Gupta R. Improvement of classification accuracy using image fusion techniques.

[9] Li S., Li Z. Effects of image fusion algorithms on classification accuracy.

[10] Subramaniam U., Subashini M. M., Almakhles D., Karthick A., Manoharan S. (2021). An expert system for COVID-19 infection tracking in lungs using image processing and deep learning techniques. *BioMed Research International*.

[11] Ganesh S. S., Kannayeram G., Karthick A., Muhibbullah M. (2021). A novel context aware joint segmentation and classification framework for glaucoma detection. *Computational and Mathematical Methods in Medicine*.

[12] Elkholy M., Hosny M. M., Farid El-Habrouk H. M. (2019). Studying the effect of lossy compression and image fusion on image classification. *Alexandria Engineering Journal*.

[13] Kumar P. M., Saravanakumar R., Karthick A., Mohanavel V. (2022). Artificial neural network-based output power prediction of grid-connected semitransparent photovoltaic system. *Environmental Science and Pollution Research 29*.

[14] Jeevanand N., Verma P. A., Saran S. (2018). Fusion of hyperspectral and multispectral imagery with regression kriging and the Lulu operators; a comparison. *The International Archives of the Photogrammetry, Remote Sensing and Spatial Information Sciences*.

[15] Chandran V., Sumithra M. G., Karthick A. (2021). Diagnosis of cervical cancer based on ensemble deep learning network using colposcopy images. *BioMed Research International*.

[16] Jiang D., Zhuang D., Huang Y., Fu J. (2011). Survey of multispectral image fusion techniques in remote sensing applications. *New Advances in Image Fusion*.

[17] Kabilan R., Chandran V., Yogapriya J. (2021). Short-term power prediction of building integrated photovoltaic (BIPV) system based on machine learning algorithms. *International Journal of Photoenergy*.

[18] Umri B. K., Wafa Akhyari M., Kusrini K. Detection of COVID-19 in chest X-ray image using CLAHE and convolutional neural network.

[19] Chandran V., Patil C. K., Manoharan A. M. (2021). Wind power forecasting based on time series model using deep machine learning algorithms. *Materials Today: Proceedings*.

[20] Kumar C. D. N., Aruna R. (2018). Contrast limited adaptive histogram equalization (Clahe) based color contrast and fusion for enhancement of underwater images. *Journal of Engineering (IOSRJEN)*.

[21] Bhan B., Patel S. (2017). Efficient medical image enhancement using CLAHE enhancement and wavelet fusion. *International Journal of Computers and Applications*.

[22] Chandran V., Patil K., Karthick A., Ganeshaperumal D., Rahim R., Ghosh A. (2021). State of charge estimation of lithium-ion battery for electric vehicles using machine learning algorithms. *World Electric Vehicle Journal*.

[23] El-Gamal F. E. Z. A., Elmogy M., Atwan A. (2016). Current trends in medical image registration and fusion. *Egyptian Informatics Journal*.

[24] Naidu V. P. S. (2012). Discrete cosine transform based image fusion techniques. *Journal of Communication, Navigation and Signal Processing*.

[25] Wang M., Shang X. (2020). A fast image fusion with discrete cosine transform. *IEEE Signal Processing Letters*.

[26] Paramanandham N., Rajendiran K. (2018). Infrared and visible image fusion using discrete cosine transform and swarm intelligence for surveillance applications. *Infrared Physics & Technology*.

[27] Zhu Z., Zheng M., Qi G., Wang D., Xiang Y. (2019). A phase congruency and local Laplacian energy based multi-modality medical image fusion method in NSCT domain. *IEEE Access*.

[28] Wang K., Zheng M., Wei H., Qi G., Li Y. (2020). Multi-modality medical image fusion using convolutional neural network and contrast pyramid. *Sensors*.

[29] Koonsanit K., Thongvigitmanee S., PT N. P. Image enhancement on digital x-ray images using n-clahe x-ray.

[30] Chavan S. S., Talbar S. N. Multimodality image fusion in frequency domain for radiation therapy.

[31] Junwu L., Li B., Jiang Y. (2020). An infrared and visible image fusion algorithm based on LSWT-NSST. *IEEE Access*.

[32] Chacko B., Agrwal S. L., Gupta S. K., Chahar H., Srivastava S. R., Srivastav N. Performance of image fusion technique using 4×4 block wavelet cosine transformation.

[33] Zhi J., Sun J., Wang Z., Ding W. (2018). Support vector machine classifier for prediction of the metastasis of colorectal cancer. *International Journal of Molecular Medicine*.

[34] Liu N., Shen J., Xu M., Gan D., Qi E. S., Gao B. (2018). Improved cost-sensitive support vector machine classifier for breast cancer diagnosis. *Mathematical Problems in Engineering*.

[35] Wang H., Shi Y., Zhou X., Zhou Q., Shao S., Bouguettaya A. Web service classification using support vector machine.

[36] Zeng X., Yuan S., Li Y., Zou Q. (2014). Decision tree classification model for popularity forecast of Chinese colleges. *Journal of Applied Mathematics*.

[37] Yang T., Song J., Li L. (2019). A deep learning model integrating SK-TPCNN and random forests for brain tumor segmentation in MRI. *Biocybernetics and Biomedical Engineering*.

[38] Siva Raja P. M., Rani A. V. (2020). Brain tumor classification using a hybrid deep autoencoder with Bayesian fuzzy clustering-based segmentation approach. *Biocybernetics and Biomedical Engineering*.

[39] Charde P. A., Lokhande S. D. (2013). Classification using K nearest neighbor for brain image retrieval. *International Journal of Scientific and Engineering Research*.

[40] Chaves R., Ramirez J., Gorriz J. M. SPECT image classification based on NMSE feature correlation weighting and SVM.

[41] Jabbar M. A., Deekshatulu B. L., Chandra P. (2013). Classification of heart disease using K-nearest neighbor and genetic algorithm. *Procedia Technology*.

[42] Guo G., Wang H., Bell D., Bi Y., Greer K. (2003). KNN model-based approach in classification. *OTM Confederated International Conferences On the Move to Meaningful Internet Systems*.

[43] Górriz J. M., Segovia F., Ramírez J., Lassl A., Salas-Gonzalez D. (2011). GMM based SPECT image classification for the diagnosis of Alzheimer’s disease. *Applied Soft Computing*.

[44] Prashanth R., Dutta Roy S., Mandal P. K., Ghosh S. (2014). Automatic classification and prediction models for early Parkinson’s disease diagnosis from SPECT imaging. *Expert Systems with Applications*.

[45] Amato G., Falchi F. KNN based image classification relying on local feature similarity.

[46] Song Y. Y., Lu Y. (2015). Decision tree methods: applications for classification and prediction. *Shanghai Archives of Psychiatry*.

[47] Mashat A. F., Fouad M. M., Philip S. Y., Gharib T. F. (2012). A decision tree classification model for university admission system. *International Journal of Advanced Computer Science and Applications*.

[48] Baranwal S. K., Jaiswal K., Vaibhav K., Kumar A., Srikantaswamy R. Performance analysis of brain tumour image classification using CNN and SVM.

[49] Nagaraj P., Muneeswaran V., Reddy L. V., Upendra P., Reddy M. V. Programmed multi-classification of brain tumor images using deep neural network.

[50] Biswas A., Islam M. S. Brain tumor types classification using K-means clustering and ANN approach.

[51] Zaw H. T., Maneerat N., Win K. Y. Brain tumor detection based on Naïve Bayes classification.

[52] Masoudi S., Mehralivand S., Harmon S. A. (2021). Deep learning based staging of bone lesions from computed tomography scans. *IEEE Access*.

[53] Welikala R. A., Remagnino P., Lim J. H. (2020). Automated detection and classification of oral lesions using deep learning for early detection of oral cancer. *IEEE Access*.

[54] Anupama M. A., Sowmya V., Soman K. P. Breast cancer classification using capsule network with preprocessed histology images.

[55] Nguyen P. T. Multiclass breast cancer classification using convolutional neural network.

[56] Erkal B., Basak S., Çiloglu A., Sener D. D. Multiclass classification of brain cancer with machine learning algorithms.

